The article "Human Brain Dynamics Reflect the Correctness and Presentation Modality of Physics Concept Memory Retrieval" was published in 2020. Journal: Front Hum Neurosci.

# Human Brain Dynamics Reflect the Correctness and Presentation Modality of Physics Concept Memory Retrieval

**DOI:** 10.3389/fnhum.2020.00331

**Published:** 2020-08-31

**Authors:** Chih-Ping Liang, Hsiao-Ching She, Li-Yu Huang, Wen-Chi Chou, Sheng-Chang Chen, Tzyy-Ping Jung

**Affiliations:** ^1^Institute of Education, National Chiao Tung University, Hsinchu, Taiwan; ^2^Department of Biology, National Changhua University of Education, Changhua, Taiwan; ^3^Institute for Neural Computation, University of California, San Diego, San Diego, CA, United States

**Keywords:** memory retrieval, physics concept, brain dynamics, presentation modality, correctness of retrieval

## Abstract

Human memory retrieval is the core cognitive process of the human brain whenever it is processing the information. Less study has focused on exploring the neural correlates of the memory retrieval of scientific concepts when presented in word and picture modalities. Fewer studies have investigated the differences in the involved brain regions and how the brain dynamics in these regions would associate with the accuracy of the memory retrieval process. Therefore, this study specifically focused on investigating the human brain dynamics of participants when they retrieve physics concepts in word vs. pictorial modalities, and whether electroencephalogram (EEG) activities can predict the correctness of the retrieval of physics concepts. The results indicated that word modality induced a significant stronger right frontal theta augmentation than pictorial modality during the physics concepts retrieval process, whereas the picture modality induced a significantly greater right parietal alpha suppression than the word modality throughout the retrieval process spurred by the physics concept presentations. In addition, greater frontal midline theta augmentation was observed for incorrect responses than the correct responses during retrieve physics concepts. Moreover, the frontal midline theta power has greater negative predictive power for predicting the accuracy of physics concepts retrieval. In summary, the participants were more likely to retrieve physics concepts correctly if a lower amount of theta were allocated during the maintaining period from 2,000 ms through 3,500 ms before making responses. It provides insight for our future application of brain computer interface (BCI) in real-time science learning. This study implies that the lower frontal midline theta power is associated with a lower degree of cognitive control and active maintenance of representations as participants approach a correct answer.

## Introduction

The memory encoding and retrieval processes are the essential cognitive processes of the human brain whenever it is processing any type of information. Memory retrieval is particularly important in determining whether or not humans can successfully retrieve the relevant information they have encoded into their long-term memory (LTM). That is whether they can reactivate and access the information stored in the LTM and make further connections among different pieces of information. If more associations or more links can be established to specific information, the information can be consolidated more efficiently and retrieved more rapidly and easily (Lang, 2000). Memory retrieval is even more pivotal for scientific learning because scientific concepts often involve a hierarchical organization, and the hierarchical level of the concepts is a crucial factor influencing the level of difficulty students experience in understanding physical concepts (She, 2004). The concepts of the higher hierarchical levels subsume more essential underlying concepts, thus making it more difficult for science learning to occur (She, 2002). Therefore, the efficiency and effectiveness of the memory retrieval of scientific concepts become critical for science learning to happen. Wilckens et al. (2012) divided retrieval into two processes: the pre-retrieval and post-retrieval processes. The pre-retrieval process can filter irrelevant information during a memory search and prepare for a retrieval attempt to occur. If the pre-retrieval processing is not sufficient, post-retrieval processing can assist in managing or refining the retrieval of contents in detail. A retrieval attempt and the post-retrieval process comprise a form of two-way processing, and a second retrieval attempt might be required before making a decision. Schacter et al. (1993) suggested that retrieval consists of the deliberate and active acquisition and accessing of past information. Heil et al. (1996, 1997) also proposed that retrieval triggers a respective pattern of neuronal activities that are the same as those occurred when the information was originally processed. Buckner and Koutstaal (1998) further divided explicit retrieval into memory search processes (attempt) and associated retrieval success (recognition or recall) processes. Bledowski et al. (2006) mentioned that retrieval contains several functional sub-processes, including stimulus evaluation, memory search, decision-making, and response organization. Previous neuroscience research regarding memory retrieval mainly studied daily-life related objects or word, whereas less research has investigated how the memory of scientific concepts is retrieved. Many physics concepts are abstract or subsume more essential underlying concepts, causing middle and high school physics to be among the most difficult subjects to learn (She, 2002, 2004; She and Liao, 2010). Thus, one of the aims of this study was to understand the brain dynamics of retrieval processes involving physics concepts in different brain regions. The results of the study may, in turn, advance our understanding of how such information is learned and processed, as well as how it is retrieved in different brain areas. Moreover, the effects of modality of presentation on human retrieving physics concepts would open a new window to facilitate students’ scientific understanding as well as advance ways of science teaching.

The article "Human Brain Dynamics Reflect the Correctness and Presentation Modality of Physics Concept Memory Retrieval" was published in 2020. Journal: Front Hum Neurosci.

Miller and Cohen (2001) suggested that the prefrontal cortex (PFC) is the main area responsible for cognitive controls including the inhibition of automatic or optimal reactions, the selection of goal orientations, the retrieval of LTM, the shifting of attention, and the monitoring and coordination of working memory (Miller and Cohen, 2001; Baddeley, 2002). Fletcher and Henson (2001), meanwhile, suggested that the frontal region is involved in the top-down control of episodic retrieval. In particular, they suggested that the ventrolateral frontal cortex manages memory search or memory retrieval from the long-term semantic memory. Cruse and Wilding (2009) reported that the PFC facilitates retrieval monitoring and assessment in the retrieval of new/old words, whereas an earlier study found that theta activation occurs in both memory encoding and retrieval tasks (Ward, 2003). Klimesch et al. (2005) suggested that frontal theta activity is closely related to enhanced attention, sustained neuronal activity, and the active maintenance of representations during the retrieval process. Theta augmentation in the forebrain during retrieval may reflect a common sign of the retrieval-related control process (Khader and Rösler, 2011). Wagner et al. (2005) reported that parietal lobe activities were observed during an episodic retrieval memory task in fMRI studies, whereas an earlier study indicated that upper alpha power increased during the processes of search and retrieval from semantic LTM (Klimesch, 1999). Freunberger et al. (2008) reported that alpha power plays an important role in the selection and coordination of the top-down control semantic retrieval process from LTM. Klimesch et al. (2007) claimed that alpha event-related desynchronization (ERD) takes part in the top-down control of the semantic operation to retain, manipulate, and retrieve the stored information. They further suggested that follow-up alpha ERS might take part in the top-down control to inhibit or block the retrieval of previous irrelevant information. In addition, the decrease of alpha power is responsible for the increment of attention, alertness, general task demands, and the processes of searching and retrieving from the LTM (Klimesch, 1999). Meyer et al. (2015) hypothesized that during sentence comprehension, the requirement of retrieval leads to frontal theta power augmentation, which is supposed to clarify the differences among stored items in verbal-working-memory retrieval. Thus, this study focused on studying both the frontal theta and parietal alpha activity during the physics concept retrieval process and aimed to better understand how different brain regions collaborate with each other to retrieve information successfully. Klimesch (1999) claimed that theta activation is stronger in good performance than in poor performance of working memory tasks. Furthermore, Klimesch et al. (2000) reported that, in comparison with correct rejections in a working memory task, target trials (i.e., remembered words) elicited stronger theta activation. Inspired by this previous work, we further sought to explore what brain regions are involved in physics concepts memory retrieval and how brain dynamics are associated with the accuracy of such retrieval.

The article "Human Brain Dynamics Reflect the Correctness and Presentation Modality of Physics Concept Memory Retrieval" was published in 2020. Journal: Front Hum Neurosci.

The aforementioned studies shed light on the potential and importance of studying which brain regions and what types of brain dynamics are associated with the memory retrieval of scientific concepts spurred by the presentation of word and pictorial stimuli. Thus, this study aimed to investigate whether and how the human brain dynamics involved in the successful memory retrieval of physics concepts are presented in different modalities (words vs. pictures). In particular, we examined oscillatory electroencephalogram (EEG) patterns during the retrieval of physics concepts presented in the picture and word forms. The objectives of this study are first, to explore whether the brain dynamics of physics concepts retrieval processing and the responsible brain regions are different when such concepts are presented in the picture vs. word modalities; second, to investigate whether the brain activities before correct and incorrect responses are different during the process of retrieving physics concepts spurred by different presentation modalities; and third, we wanted to explore whether EEG activities can be used to predict the correctness of the retrieval of physics concepts.

## Materials and Methods

### Subjects

A total of 51 undergraduate students (29 males, 22 females) aged 18–22 years participated in the study. All of the participants were right handed and had a normal or corrected-to-normal vision. They were informed about the experiment procedure, read and signed a consent form, and paid for their participation. The Institutional Review Board of the China Medical University Hospital approved this study. All of the students who volunteered to take part in the study majored in science and had learned the physics concepts used in the present study in high school. After EEG pre-processing, four participants’ EEG data were excluded from further analysis because they contributed fewer than two independent components to the component clusters. That is, the EEG data from only 47 of the 51 participants (26 males, 21 females) were used in the study.

The article "Human Brain Dynamics Reflect the Correctness and Presentation Modality of Physics Concept Memory Retrieval" was published in 2020. Journal: Front Hum Neurosci.

### Experiment and Procedure

To explore the cognitive process of the retrieval of physics concepts presented in different modalities, 90 physics concepts items related to the topics of mechanics, optics, electromagnetics, and thermodynamics were selected from secondary school physics textbooks and presented either in pictorial modality (45 physics concept items) or word modality (45 physics concept items). For the picture modality, each trial started with an 800-ms fixation, followed by a 2,000-ms presentation of the physics concept item, a 2,000-ms blank, and then a “go” signal. Each subject had to provide an oral response as soon as possible after the go signal was presented on the monitor, and each trial lasted a total of 6.8 s. Figure 1A shows a sample pictorial trial of synchromesh gears, which requires the participants to retrieve the concept of synchromesh gears from their LTM and make a verbal response. For the word modality/representation, each trial lasted 8.8 s, with all the parameters being the same as in the picture representation except that the presentation of each physics concept definition lasted for 4,000 ms. Figure 1B shows a sample trial of the definition of power was presented in word (text), which requires the participants to retrieve the concept of power from their LTM and make a verbal response. The responses of the participants were recorded, and the correctness of their responses was analyzed after the data collection. For each modality, three out of the 45 items were first presented as a practice before the formal experiment.

**Figure 1:** The retrieval stimuli of physics concepts are presented in the picture and word modalities. **(A)** Sample trial of synchromesh gears is presented in picture for 2,000 ms, followed by a 2,000-ms blank for the participants to retrieve the concept, and then make a verbal response as soon as they see a “go” signal. **(B)** Sample trial of the definition of power is presented in word (text) for 4,000 ms, followed by a 2,000-ms blank for the participants to retrieve the concept, and then make a verbal response as soon as they see a “go” signal.

The article "Human Brain Dynamics Reflect the Correctness and Presentation Modality of Physics Concept Memory Retrieval" was published in 2020. Journal: Front Hum Neurosci.

### Data Collection

In this study, all 42 trials of the physics concepts in each modality were presented by the STIM2 software, and EEG data from each participant were recorded continuously with a Neuroscan SynAmps2 amplifier (Neuroscan, El Paso, TX, USA) with 66 electrodes mounted in an elastic cap. The EEG signals were filtered using an analog band-pass filter from 0.01 to 100 Hz, and the sampling rate was 1,000 Hz. Inter-electrode impedance was maintained below 5 kΩ. The electrode locations followed the international 10-20 system, and all the electrodes were referenced to the linked mastoids. Four separate bipolar electrodes recorded the vertical (vEOG) and horizontal (hEOG) eye movements.

### EEG Data Analysis

The recorded EEG data were first digitally band-pass filtered using the EEGLAB toolbox (Delorme and Makeig, 2004) between 0.5 and 50 Hz and down-sampled to 250 Hz. After the EEG data pre-processing, the EEG data were submitted to extended independent component analysis with information maximization (Infomax; Lee et al., 2000) using the runica function in the EEGLAB toolbox (Makeig et al., 1997). In this study, the runica training parameters of stopping weight change were set to 1e^−7^ or 1e^−8^. The fast Fourier transformation was then used to transform the EEG activities into power spectrum density in the following frequency bands: θ (4–7.9 Hz), α (8–12.9 Hz), and low β (13–18 Hz).

### Component Selection

All the resultant independent components (ICs) were characterized into brain or non-brain components. We then used the boundary element head model, as implemented in the DIPFIT toolbox (Oostenveld and Oostendorp, 2002), to calculate the equivalent current dipole model for each of the selected brain components. The ICs with bilaterally distributed scalp maps were fitted with a dual equivalent dipole model with a positional symmetry constraint. Only the ICs with equivalent dipole models accounting for more than 85% of the actual IC scalp map variance and the ICs with an equivalent dipole model located inside the head sphere were included in the further analysis.

### Independent Component Clustering

Before clustering, the component spectrum power, event-related potential (ERP), event-related spectral perturbation analysis (ERSP), inter-trial coherence, and scalp topography of each independent component were computed. With the exception of the dipole source location that was featured in only three dimensions (*x*, *y*, *z*), other measures were compressed into a 10-dimension vector, resulting in a 53-dimensional feature space. Each IC with a 53-dimensional cluster position vector was further compressed by principal component analysis into a 10-dimensional vector. To normalize the variance from the different measures in the cluster position vector, the dipole location was given a weight of 20, ERSP was given a weight of 9, and other measures (spectrum, ERP, inter-trial coherence, and scalp topography) were given a weight of 1. Any ICs whose distance to the cluster centroid was greater than three standard deviations away from the cluster centroid were removed. The K-means clustering algorithm, a particular modeling technique involving the grouping of homogeneous ICs across subjects by taking various measures of spectra, ERP, ERSP, inter-trial coherence, and scalp topography and dipole location, was used to group the ICs into 42 clusters (with only three dimensions). Subsequently, visual inspection was applied to remove improper ICs from each cluster according to their dipole locations, ERSPs, scalp maps, and power spectra.

The article "Human Brain Dynamics Reflect the Correctness and Presentation Modality of Physics Concept Memory Retrieval" was published in 2020. Journal: Front Hum Neurosci.

### Event-Related Spectral Perturbation

The component activations of each IC within a component cluster were divided into non-overlapping epochs of 7.5 and 9.5 s for the picture and word trials, which included the duration from 1,000 ms before the presentation onset to 2,500 ms after the go signal. The IC activations for each trial were then transformed into a spectrographic image (event-related spectral perturbation, ERSP) using three-cycle Morlet wavelets in a frequency range between 3 and 50 Hz (Makeig, 1993) implemented in the EEGLab. The ERSP was used to visualize the mean event-related spectral power changes of the selected clusters over time relative to an experimental event. Calculating an ERSP requires averaging the power spectra across all the trials of the ICs within each cluster. Then, the ERSP results are plotted as relative spectral log amplitudes from the baseline on a 2D time–frequency plane with the different colors representing different power values (Makeig, 1993; Delorme and Makeig, 2004; e.g., Figures 2D–I, 3B,C,E,F). This study uses bootstrap testing to examine the statistical significance of the baseline-corrected spectral differences between two conditions (e.g., word and picture representations in Figures 2J,L,N, correct and incorrect responses in Figures 3D,G). Specifically, we constructed surrogate data by repetitively shuffling spectral estimates between two conditions (e.g., correct and incorrect trials) and re-computing the spectral differences using the shuffled data. We repeated the process 200 times, resulting in a surrogate difference distribution whose specified percentiles are taken as significance thresholds. Then, we test if the original spectral difference between the two conditions is in the tail of the surrogate difference distribution. Under the null hypothesis of no difference between the conditions, the original difference should not be in the tail. If it is, we can assess the probability of rejecting the null hypothesis (Delorme and Makeig, 2004). This study also explores the temporal dynamics of the EEG spectra under different conditions (e.g., word and picture representations, correct and incorrect responses). We aggregate the time-series of the theta and alpha power across subjects and then use *t*-test to examine if the spectral differences between the two conditions are statistically significant at each time point after stimulus presentation (Figures 2K,M,O, 3H–K).

The article "Human Brain Dynamics Reflect the Correctness and Presentation Modality of Physics Concept Memory Retrieval" was published in 2020. Journal: Front Hum Neurosci.

**Figure 2:** The right frontal, right parietal, and right occipital clusters. **(A–C)** Scalp maps and dipole locations. **(D–I)** Event-related spectral perturbation analysis (ERSP’s) for word trials and picture trials. **(J,L,N)** The bootstrap statistics indicating significant (*p* < 0.01) power changes between the word and picture conditions. **(K,M,O)** Mean spectral comparison between the word and picture conditions in the theta band or alpha band; green represents the mean power of word trials, purple represents the mean power of picture trial.

**Figure 3:** The frontal midline clusters. **(A)** Scalp map and dipole location. **(B,C)** ERSP’s comparison between the incorrect and correct responses to picture trials. **(D)** The bootstrap statistics indicating significant (*p* < 0.01) power changes between the incorrect and correct responses for the picture trials. **(E,F)** ERSP’s comparison between the incorrect and correct responses for the word trials. **(G)** The bootstrap statistics indicating significant (*p* < 0.01) power changes between the incorrect and correct responses for word trials. **(H,I)** Mean spectral comparison between the incorrect and correct responses in the theta band and alpha band; blue represents the incorrect response, red means the correct response for picture trial. **(J,K)** Mean spectral comparison between the incorrect and correct responses in the theta band and alpha band; blue represents the mean power of incorrect responses, red represents the mean power of correct response for the word trials. Note: subplots **(H–K)** miss the bottom part of the figure and X-tick labels.

## Results

### The Associations of EEG Dynamics With the Physics Concepts Retrieval Process

The right frontal, left frontal, right parietal, left parietal, right occipital, and left occipital cluster recruited 27, 34, 30, 29, 28, and 30 independent components from 27, 34, 30, 29, 28, and 30 subjects (out of 45 subjects), respectively. The ERSP was employed to visualize the mean event-related spectral changes of the selected clusters over time, which showed the neural activities in the right hemisphere were very similar to those in the left hemisphere. However, the activities in the right hemisphere were considerably stronger than those in the left hemisphere; thus, the following results specifically focus on the right hemisphere.

The article "Human Brain Dynamics Reflect the Correctness and Presentation Modality of Physics Concept Memory Retrieval" was published in 2020. Journal: Front Hum Neurosci.

The average scalp maps and the dipole locations of the clusters in the right frontal cluster are shown in Figure 2A. The results of the right frontal average ERSP image (Figures 2D,E) and ERSP transforms (Figure 2K) showed that the theta band power increased after the stimulus onsets, with the power activation being maintained across the entire physics concept retrieval process until the go signal, regardless of the word or picture presentation modality. The bootstrap analysis of the picture and word modalities in the right frontal region showed that theta power was significantly stronger for the word modality than that for the picture modality marked in red color (*p* < 0.01; Figure 2J). The ERSP of the right parietal cluster showed that the alpha power in the picture modality was suppressed more than that in the word modality during the retrieval process, including the concept presentation and maintenance periods (Figures 2B,F,G). Both the bootstrapping and ERSP analyses indicated that the picture modality showed significantly more alpha suppression than the word modality during the retrieval process (Figures 2L,M). For the right occipital cluster, the theta power increased sharply after the onsets of the physics concept stimulus presentation, followed by an alpha suppression, in both the picture and word modalities (Figures 2C,H,I). The theta augmentation and alpha suppression were maintained until the end of each physics concept presentation for both the picture and word modalities. The bootstrapping and ERSP analyses indicated that the picture modality induced a significantly greater alpha suppression than the word modality throughout the retrieval process spurred by the physics concept presentations (Figures 2N,O).

### Frontal Midline Theta and Alpha Correlates of the Successful Retrieval of Physics Concepts

We next investigate the associations between the EEG spectra and task performance and found that the frontal midline cluster revealed greater theta power and alpha power in the incorrect trials (Figure 3B) than in the correct trials (Figure 3C). Both bootstrapping and ERSP analyses showed significantly greater theta and alpha power augmentation in the incorrect responses than in the correct responses at the frontal midline cluster (*p* < 0.01) during the entire retrieval process, including the stimulus presentation and retrieval stages (Figures 3D,H,I).

The article "Human Brain Dynamics Reflect the Correctness and Presentation Modality of Physics Concept Memory Retrieval" was published in 2020. Journal: Front Hum Neurosci.

A comparison of the response accuracy (incorrect vs. correct) of the physics concept retrieval for the word presentations showed that the ERSP of the frontal midline cluster exhibited a greater theta power increase in the incorrect responses than in the correct responses (Figures 3E,F). In addition, both the bootstrapping and ERSP analyses revealed greater theta augmentation in the incorrect trials than in the correct trials (*p* < 0.01; Figures 3G,J,K).

### Frontal Midline Theta and Alpha Power Predict the Accuracy of the Memory Retrieval of Physics Concepts Spurred by Pictorial Stimuli

The results of the ERSP and the power mean plots in Figure 3 showed that the distinct spectral patterns between the correct and incorrect trials mainly exhibited in the frontal midline cluster; thus, we further conducted a correlation analysis between the spectra of the frontal midline cluster and the corresponding retrieval performance (i.e., correct vs. incorrect responses; Figures 4A,B). Figure 4B shows that for physics concepts presented in the pictorial form, the theta and alpha power between 2,000 and 3,500 ms was negatively correlated with the accuracy of retrieval performance. Based on the ERSP and correlation results, this study further performed a logistic regression analysis to explore whether the frontal theta and alpha power could predict subjects’ retrieval physics concepts accuracy. In this case, the dependent nominal is correct/incorrect response and the independent measurements are theta and alpha power, respectively. Table 1 shows that the frontal midline theta (5 Hz) power had a negative influence on students’ likelihood of accurately responding to the retrieval physics concepts during the period from 2,000 to 3,500 ms [x-standardized coefficient (βSx) = −2.2916 (5 Hz), *p* < 0.001]. Figure 5A presents the plot of the natural logarithm of estimated odds for response accuracy as a blue line according to the SD of the frontal midline theta power. A 1-SD decrease in the frontal midline theta power was accompanied by a 2.2916 increase in the log odds of responding correctly. Figure 5C presents the percentage of predicted probability for correct responses according to the power of the frontal midline theta in the blue curve. The predicted probability of a correct response was greater than 89.53% when the frontal theta power was lower than 0 dB (see the red line), and the predicted probability of correct response was close to 100% when the frontal theta power was lower than −1 dB (see the edge of the red line that intersects the blue curve). The predicted probability of correct answer was higher than 86.45% when the frontal midline theta power was lower than 0.12 dB (see the intersecting point of the red line and green line; red line: only correct responses were observed when the frontal midline theta power was lower than 0.12 dB). This result indicates that the students were more likely to retrieve physics concepts correctly if they had less theta augmentation during the period from 2,000 through 3,500 ms. In addition, Table 2 shows that the frontal alpha 10 Hz power had a negative influence on the likelihood of accurately responding to the retrieval physics concepts during the period from 2,000 to 3,500 ms [x-standardized coefficient (βSx) = −0.8169 (5 Hz), *p* < 0.001]. Figure 5B indicated that a 1-SD decrease in the frontal midline alpha power was accompanied by a 0.8169 increase in the log odds of responding correctly. Figure 5D further showed that the predicted probability of correct response was greater than 73.58% when the frontal alpha power was lower than 0 dB (see the red line), and that the predicted probability of correct response was around 92.54% when the frontal alpha power was lower than −1.48 dB (see the edge of the red line and blue curve). The predicted probability of a correct answer was about 85.65% when the frontal midline theta power was lower than −0.76 dB (see the intersecting point of the red line and green line; red line: only correct responses were observed when the frontal midline theta power was lower than −0.76 dB). That is, the students were more likely to respond correctly if they had less alpha augmentation during the period of 2,000–3,500 ms. In sum, compared with the frontal midline alpha, the frontal midline theta power was a better predictor of participants’ retrieval physics concepts according to both results of the natural logarithm of estimated odds for response accuracy and the percentage of predicted probability for correct responses.

The article "Human Brain Dynamics Reflect the Correctness and Presentation Modality of Physics Concept Memory Retrieval" was published in 2020. Journal: Front Hum Neurosci.

**Figure 4:** Correlations between electroencephalogram (EEG) spectrum and subject response (correct vs. incorrect) for the frontal midline cluster. Correlation plots show the correlations between EEG spectrum and subject response (correct vs. incorrect) in the time windows of the **(A)** word modality from −200 to 8,100 ms and **(B)** picture modality from −200 to 6,500 ms.

**Table 1:** Analytic results of electroencephalogram (EEG) power spectra over time in the frontal midline cluster, using a logistic regression model (5 Hz).

Covariate	2,000–3,500 ms				
	b	bstdx	bstdy	bstdxy	*p*-value
Theta (5 Hz)	−2.44472	−2.2916	−0.8365	−0.7841	<0.001

*b, raw coefficient; bstdx, x-standardized coefficient; bstdy, y-standardized coefficient; bstdxy, fully standardized coefficient*.

**Figure 5:** **(A,B)** The plots show the estimated odds of the response accuracy according to the standard deviation of the frontal midline theta (5 Hz; **A**) and alpha 10 Hz power **(B)** across trials. **(C,D)** The plots show that the predicted probability of correct responses (blue color) according to the frontal midline theta 5 Hz **(C)** and alpha 10 Hz power **(D)** across trials in blue color. The observed correct and incorrect responses are presented in red and green color, respectively.

**Table 2:** Analytic results of EEG power spectra over time in the frontal midline cluster, using a logistic regression model (10 Hz).

Covariate	2,000–3,500 ms				
	b	bstdx	bstdy	bstdxy	*p*-value
Alpha (10 Hz)	−1.01650	−0.8169	−0.5110	−0.4107	<0.001

*b, raw coefficient; bstdx, x-standardized coefficient; bstdy, y-standardized coefficient; bstdxy, fully standardized coefficient*.

## Discussion

### The Associations of EEG Dynamics With the Physics Concepts Retrieval Process

The study results demonstrated that the retrieval of physics concepts spurred by both the pictorial and word modalities elicited strong theta power in the right frontal region across the entire physics concept retrieval stage until the presentation of the go signal. Previous studies also reported that a strong increase in theta oscillations during the working memory task and that the increased theta activity was sustained during the retention period until information had been retrieved (Raghavachari et al., 2001; Lai et al., 2012; She et al., 2012; Huang et al., 2013; Chou et al., 2015). Klimesch et al. (2005) reported that either the maintenance of information in the short-term memory or the execution of control processes such as rehearsal was reflected by a sustained theta-power increase. Other studies also reported that theta oscillations are involved in the active maintenance and recall of working memory representations (Kahana et al., 1999; Jensen and Tesche, 2002). These results suggested that the frontal region is responsible for maintaining the information to be processed in the working memory until the information has been retrieved successfully. Our results also indicated that the theta power was significantly stronger for the word modality than for the picture modality during the retrieval of physics concepts, which is in line with the results of a previous encoding study (Lai et al., 2012). Our study provides new evidence that the frontal theta activity during the retrieval process shares similar EEG patterns to those of the encoding process reported by previous studies.

The results also showed that the right parietal region exhibited significantly more alpha suppression during the retrieval of the pictorial presentations of physics concepts when compared with the word presentations. Klimesch (1999) pointed out that lower alpha suppression represents attentional demands, whereas upper alpha suppression is reflected in the processes of searching and retrieving information from the semantic LTM. Freunberger et al. (2008) found that semantic information retrieval from the LTM can cause an upper alpha decrease, which reflected the semantic access instead of the task difficulty. They also mentioned that alpha played an important role in the selection and coordination of the top-down control of LTM. Other studies found that the parietal lobe is responsible for the capacity limit of the short-term memory (Postle and Awh, 2004) or memory load (Vogel and Machizawa, 2004). Wagner et al. (2005) pointed out that the parietal lobe is an interface linking the PFC (executive) and the medial temporal area (LTM—declarative). Furthermore, another fMRI study has reported that parietal lobe activation was observed during the performance of an episodic memory retrieval task (Wagner et al., 2005). Relatedly, there are three possible hypotheses regarding the role of the parietal lobe in the retrieval of episodic memory. The first is that it serves as an output buffer, which is analogous to the episodic buffer hypothesis proposed by Baddeley (2002). The second is that it acts as a signal to increase memory strength and enhances the degree of the activation for final decision-making. The third is that it provides attention to memory, including in the superior parietal cortex and the inferior parietal cortex, to help the top-down and bottom-up control of memory (Wagner et al., 2005; Simons and Mayes, 2008).

The article "Human Brain Dynamics Reflect the Correctness and Presentation Modality of Physics Concept Memory Retrieval" was published in 2020. Journal: Front Hum Neurosci.

In addition, our findings also revealed that the occipital theta power increases sharply after the onsets of either word or pictorial presentations of physics concepts, which is followed by a marked alpha suppression. This finding is consistent with those of previous studies (Lai et al., 2012; She et al., 2012; Huang et al., 2013; Chou et al., 2015). Moreover, our results indicated that the picture modality induced a significantly greater alpha suppression than the word modality throughout each physics concept presentation for both the right parietal and the right occipital areas. Alpha power often decreases in tasks requiring greater demands and cognitive effort, primarily at the posterior sites (Gevins et al., 1997). Huang et al. (2013) showed that the posterior (central parietal and occipital) theta oscillation peaked at around 200 ms after stimulus onsets. They speculated that the posterior theta might be driven by a combination of the following: (1) sensory processing; (2) theta gating; and (3) stimulus selection. Klimesch et al. (2011) proposed that sensory information is processed for up to 100 ms after a stimulus onset, which allows for an early categorization for the encoded stimulus. Klimesch et al. (2011) also suggested that the posterior alpha activity may reflect a specific type of attention, which controls the flow of information into and out of the LTM, and that it helps to narrow down the relevant search area in the memory. Huang et al. (2013) suggested that the posterior alpha ERD might be associated with stimulus recognition and the control of the flow of information into and out of the LTM.

### Frontal Midline Theta and Alpha Power Predicts the Successful Retrieval of Physics Concepts

The study results also indicated that the frontal midline cluster revealed a significantly greater theta power and alpha power in the incorrect trials than in the correct trials for both the word and pictorial modalities. In addition, the results of the correlational analysis of the picture modality revealed that the frontal midline theta and alpha power from 2,000 to 3,500 ms was negatively correlated with the correctness of the retrieval performance. In short, the higher the frontal midline theta power, the more likely the subjects were to make an incorrect response in the picture modality. Moreover, the logistic regression analysis further demonstrated that both theta power and alpha power had a negative impact on the students’ likelihood of accurately retrieving physics concepts. The students were more likely to retrieve physics concepts correctly if a lower amount of theta and alpha power were allocated during the maintaining period from 2,000 ms through 3,500 ms before making responses. The natural logarithm of estimated odds and predicted probability of retrieving physics concepts increased when the frontal midline theta and alpha power decreased. Compared with the frontal midline alpha, the frontal midline theta power was a better predictor of participants’ retrieval physics concepts. Klimesch et al. (2005) have suggested that frontal theta is involved with the execution of cognitive control, such as shift and enhanced attention or rehearsal. Other studies have suggested that the frontal theta activity was closely related to enhanced attention, sustained neuronal activity, and the active maintenance of representations during encoding and retrieval (Raghavachari et al., 2001; Jensen and Tesche, 2002; Gevins and Smith, 2003). Our findings demonstrated that the lower frontal midline theta power, the more likely of the correct physics concepts they can retrieve. The aforementioned studies provide the support that the lower frontal midline theta power may result in a lower degree of cognitive control and the maintenance of working memory information as participants approach the correct answer. On the other hand, Metcalfe and Wiebe (1987) investigated the feelings of warmth reported by participants when solving algebra problem and their results indicated that distinct incremental increases in feelings of warmth were observed as the participants approached solutions to the problems. Our results further advanced Metcalfe and Wiebe’s (1987) findings to speculate that the lower frontal midline theta power is not only correlated with lower degrees of cognitive control and the maintenance of working memory information but that it is also correlated with the warmer feelings of participants as they approach the correct answers.

The article "Human Brain Dynamics Reflect the Correctness and Presentation Modality of Physics Concept Memory Retrieval" was published in 2020. Journal: Front Hum Neurosci.

When retrieving physics concepts presented in a pictorial modality, the participants exerted more mental effort to generate incorrect answers than correct answers and to maintain the operation of the retrieval of the physics concepts in the working memory. Our results supported the previous conflict-monitoring theory, which suggests that the timing of the ACC activations reflects that conflicts for correct and incorrect responses should differ (Botvinick et al., 2004; Krug and Carter, 2010) and a previous study of EEG oscillations reported pronounced differences between correct and incorrect decision-making in the ACC cluster (Huang et al., 2018). This current study not only confirms that such ACC oscillations have the ability to predict the correctness of responses but also provides compelling evidence that the frontal midline theta and alpha power during the maintenance period has the negative predictive power to predict the accuracy of the retrieval of physics concepts. In short, the participants were more likely to retrieve physics concepts correctly if a lower amount of theta were allocated during the maintaining period from 2,000 ms through 3,500 ms before making responses. These results would benefit our future application of brain computer interface (BCI) in real-time science learning.

## Data Availability Statement

The raw data supporting the conclusions of this article will be made available by the authors, without undue reservation.

## Ethics Statement

The studies involving human participants were reviewed and approved by the Institutional Review Board China Medical University Hospital/DMR100-IRB-221. The patients/participants provided their written informed consent to participate in this study.

## Author Contributions

H-CS: conceptualization. C-PL, H-CS, L-YH, W-CC, and S-CC: design and methodology. L-YH, W-CC, and S-CC: data collection. C-PL: data analysis. H-CS: supervision. H-CS, C-PL, L-YH, and T-PJ: validation. H-CS, C-PL, L-YH, and T-PJ: writing—reviewing and editing.

The article "Human Brain Dynamics Reflect the Correctness and Presentation Modality of Physics Concept Memory Retrieval" was published in 2020. Journal: Front Hum Neurosci.

## Conflict of Interest

The authors declare that the research was conducted in the absence of any commercial or financial relationships that could be construed as a potential conflict of interest.
